# Restoration of High Frequency Auditory Perception After Robot-Assisted or Manual Cochlear Implantation in Profoundly Deaf Adults Improves Speech Recognition

**DOI:** 10.3389/fsurg.2021.729736

**Published:** 2021-09-10

**Authors:** Renato Torres, Hannah Daoudi, Ghizlene Lahlou, Olivier Sterkers, Evelyne Ferrary, Isabelle Mosnier, Yann Nguyen

**Affiliations:** ^1^Unité Fonctionnelle Implants Auditifs, Service Oto-Rhino-Laryngologie, AP-HP/Sorbonne Université, Paris, France; ^2^Centre de Recherche en Audiologie Adulte, GHU Pitié-Salpêtrière/Fondation Pour l'Audition, AP-HP, Paris, France; ^3^Technologies et Thérapie Génique Pour la Surdité, Institut de l'Audition, Institut Pasteur, INSERM, Paris, France; ^4^Departamento de Ciencias Fisiológicas, Facultad de Medicina, Universidad Nacional de San Agustín de Arequipa, Arequipa, Peru

**Keywords:** ear surgery, hearing loss, translocation, pure-tone audiometry, hearing performance, hearing outcomes

## Abstract

**Background and Purpose:** Robot-assisted cochlear implantation has recently been implemented in clinical practice; however, its effect on hearing outcomes is unknown. The aim of this preliminary study was to evaluate hearing performance 1 year post-implantation whether the electrode array was inserted manually or assisted by a robot.

**Methods:** Forty-two profoundly deaf adults were implanted either manually (*n* = 21) or assisted by a robot (RobOtol®, Collin, Bagneux, France) with three different electrode array types. Participants were paired by age, and electrode array type. The scalar position of the electrode array in the cochlea was assessed by 3D reconstruction from the pre- and post-implantation computed tomography. Pure-tone audiometry and speech perception in silence (percentage of disyllabic words at 60 dB) were tested on the implanted ear 1 year post-implantation in free-field conditions. The pure-tone average was calculated at 250–500–750 Hz, 500–1,000–2,000–3,000 Hz, and 3,000–4,000–8,000 Hz for low, mid, and high frequencies, respectively.

**Results:** One year after cochlear implantation, restoration of the high-frequency thresholds was associated with better speech perception in silence, but not with low or mid frequencies (*p* < 0.0001; Adjusted *R*^2^ = 0.64, polynomial non-linear regression). Although array translocation was similar using either technique, the number of translocated electrodes was lower when the electrode arrays had been inserted with the assistance of the robot compared with manual insertion (*p* = 0.018; Fisher's exact test).

**Conclusion:** The restoration of high-frequency thresholds (3,000–4,000–8,000 Hz) by cochlear implantation was associated with good speech perception in silence. The numbers of translocated electrodes were reduced after a robot-assisted insertion.

## Introduction

Cochlear implants are medical devices aiming to electrically stimulate ganglion of the auditory nerve and to restore hearing in patients with severe to profound hearing loss. The hearing outcomes after cochlear implantation depend on improvable (e.g., electrode array insertion, technological advances of array/processor), and definite factors (e.g., age at implantation, duration of preoperative profound deafness, etiology of the hearing loss).

Electrode array insertion is performed surgically with micro-instruments under microscopic view. Optimization of this surgical step has been associated with hearing outcomes, and aims to insert the electrode array into the scala tympani (1–4), and to avoid, whenever possible, damage to the basilar membrane to preserve residual hearing when acoustic stimulation of the higher turns of the cochlea is possible (5). For this purpose, there is growing interest in using robots for cochlear implantation with different approaches such as direct external access to the cochlea (6, 7), using a teleoperated robot to insert the electrode array (8–10), and coupling robot and navigation to correctly align the electrode array with the insertion axis (11, 12). A robot overcomes the inaccuracy of manual insertion, and presumably allows cochlear trauma to be reduced during electrode array insertion (10). However, hearing outcomes after robot-assisted cochlear implantation remain to be analyzed and compared to those obtained after manual cochlear implantation.

With regard to speech perception in cochlear implanted patients, its relationship with restoration of post-implantation pure-tone thresholds is not clear. Some studies show that pure-tone performance is not related to speech perception (13). On the other hand, preservation of low-frequency auditory hearing is associated with better speech perception after cochlear implantation (14). However, in non-implanted patients, a deterioration of the speech perception is associated with an impairment of the mid and high-frequency thresholds (15).

The aim of the study was to assess speech perception in silence 1 year postoperatively in profoundly deaf adults who underwent robot-assisted or manual cochlear implantation, and its relationship with restoration of pure-tone audiometry.

## Materials and Methods

### Patients

This is a retrospective study that included 42 patients who underwent cochlear implantation in a tertiary referral center. All patients give their consent to participate in the study, and the protocol was approved by the Institutional Review Board–CNIL N° 20191219182243. Two groups were established according to the electrode array insertion technique: robot-assisted (*n* = 21) or manual (*n* = 21). Each patient from the robot-assisted group was paired with one of the manually inserted group by age, and cochlear implant type. Robot-assisted cochlear implantations were performed between July 2019 and March 2020, and between July 2018 and November 2019 for manual implantation. Data on the electrode array position have been partially published (17 cases from the robot-assisted group and 21 cases from the manually inserted group) (10). All patients had no residual hearing before the surgery and underwent hearing tests 1 year after surgery.

### Cochlear Implant

Three types of electrode arrays were inserted:

- Cochlear™ Nucleus® CI522 or CI622 (Cochlear, Lane Cove, Australia) (*n* = 22). This is a straight electrode array with an active length of 19.1 mm and 22 electrodes;
- Advanced Bionics HiFocus™ Slim J (Advanced Bionics, Valencia, CA, USA) (*n* = 16). This is a straight electrode array with an active length of 20 mm and 16 electrodes;
- Advanced Bionics HiFocus™ Mid-Scala electrode array (*n* = 6). This pre-curved electrode array has an active length of 15.5 mm and 16 electrodes.

### Robot Assisted and Manual Electrode Array Insertion

All surgical procedures were performed by two senior surgeons (IM and YN). A classical surgical approach was used to reach the round window region: retroauricular incision, mastoidectomy, and posterior tympanotomy. The array was usually inserted through the round window except in two cases in whom a cochleostomy was performed due to a non-visible round window.

With regard to the robot-assisted insertions, the RobOtol® arm (Collin, Bagneux, France) was controlled by the surgeon using a SpaceMouse® (3DConnexion, Waltham, MA, USA). For straight arrays, insertion was completely performed at a speed of 0.25 mm/s with specifically designed insertion tools (Collin, Bagneux, France; Cochlear CI522/622: RBT-2302, and AB SlimJ: RBT-2301). The Mid-Scala array was positioned on the insertion tool and both were coupled to the robot arm (Collin, Bagneux, France; AB Mid-Scala: RBT-0406). The array was partially inserted up to the mark indicating the beginning of the coiling of the basal turn and then manually ejected from the insertion tool. With regard to the manual insertions, they were performed using surgical instruments specially designed by the manufacturer.

### Radiological Analysis

Pre-implantation computed tomography (CT) was performed in all patients. Distance A (from the center of the round window and the lateral wall at 180° passing through the modiolus), and distance B (perpendicular to distance A from the lateral wall at 90° and 270° and passing through the modiolus) were determined using 3D multiplanar reconstruction of the images performed using Horos v.2.2.0 open source software (https://horosproject.org/). Post-implantation CT was performed 24 h after surgery. Using the same 3D multiplanar reconstruction, the number of extracochlear electrodes, and the depth of insertion (measured in degrees from the line between the center of the round window and the modiolus and the most apical electrode) were determined.

Three-dimensional reconstruction models were obtained using ITK-SNAP v.3.4.0 (http://www.itksnap.org). This method was used to determine the intrascalar position of each electrode according to the basilar membrane as previously described (10) and validated with microscopy analysis (16). 3D reconstructions of the semicircular canals and the basilar membrane were obtained from the pre-implantation CT images. 3D reconstructions of the semicircular canals and the electrode array were obtained from the post-implantation CT. The fusion of both pre- and post-implantation 3D models was achieved automatically based on the orthogonal position of the semicircular canals using CloudCompare v.2.10.2 GPL software (http://www.cloudcompare.org/) (Figure 1).

**Figure 1:** Example of top **(A)**, bottom **(B)**, and lateral **(C)** views of the basilar membrane to assess the position of each electrode in relation to the basilar membrane. The positions of the basilar membrane and semicircular canals were obtained from the pre-implantation computed tomography (CT) (in green). The positions of the electrode array and semicircular canals were obtained from the post-implantation CT (in red). Both models were automatically merged according to the position of the semicircular canals that were not modified by the artefact of the electrode array. In this example, the electrode array was below the basilar membrane and consequently fully inserted into the scala tympani (no array translocation).

The position of each electrode was determined according to its position relative to the basilar membrane as either a non-translocated electrode (under the basilar membrane) or a translocated electrode (above the basilar membrane). Array translocation was defined when at least one electrode was located in the scala vestibuli. The location of the translocation was determined according to the baseline (0° degrees) between the center of the round window and the modiolus and classified as proximal (start of array translocation before 180°), or distal (after 180°). The percentage of translocated electrodes was calculated as the number of translocated electrodes/total number of electrodes in the array × 100.

### Evaluation of Hearing Performance

Hearing tests were performed 1 year after surgery. The implanted ear was independently assessed in an acoustically isolated room, without any hearing aid on the contralateral side and the ear plugged if necessary. The speaker was placed 1 meter in front of the patient. Free-field pure-tone audiometry was assessed to determine the hearing thresholds at the frequencies 250, 500, 750, 1,000, 2,000, 3,000, 4,000, and 8,000 Hz. Based on the Committee on Hearing and Equilibrium guidelines, the pure-tone average (PTA) was calculated as the mean of the thresholds at 500, 1,000, 2,000, and 3,000 Hz (17). From this interval, a low-frequency PTA (250–500–750 Hz) and a high-frequency PTA (3,000–4,000–8,000 Hz) were calculated.

Speech perception in silence was assessed using disyllabic words and the speech discrimination score (SDS) was determined at 60 dB SPL and expressed as the percentage of words correctly recognized at this acoustic pressure.

### Statistical Analysis

All numeric variables were expressed as means and standard deviations. Non-parametric tests were performed to assess the association between hearing performance and robotic/manual insertion and the intrascalar position of the electrode array. Linear and non-linear regression were performed to analyze the association between speech perception in silence and pure-tone audiometry threshold. The models were compared using ANOVA analysis to choose the best fitted model. All statistical analysis was performed using R v3.3.3 statistical software (https://www.R-project.org/). A *p* < 0.05 was considered to be significant.

## Results

### Hearing Performance and Electrode Array Insertion Technique

Pre-implantation clinical data from the patients are shown in Table 1. There was no difference in speech perception in silence between robot-assisted and manual electrode array insertion techniques (Table 2). Regarding the pure-tone thresholds, again similar results were observed between robot and manual insertion techniques for low-, mid-, and high-frequency PTA (Table 2).

**Table 1:** Clinical characteristics of the implanted patients.

**Patient characteristics**	**Robot-assisted insertion (** ***n*** **= 21)**	**Manual insertion (** ***n*** **= 21)**
Age (years)	57 ± 20.8 [21–86]	54 ± 1.6 [22–82]
Sex: M/F	(8), 38%/(13), 62%	(10), 48%/(11), 52%
Duration of deafness (years)	23 ± 11.5 [4–45]	24 ± 17.3 [4–64]
Preoperative PTA–implanted ear (dB)	114 ± 11.9 [95–120]	111 ± 16.3 [89–120]
Preoperative SDS–implanted ear (%)	0 ± 0	0 ± 0
Preoperative PTA–non-implanted ear (dB)	93 ± 18.5 [64–120]	102 ± 18.2 [59–120]
Preoperative SDS–non-implanted ear (%)	1 ± 3.2 [0–10]	3 ± 8.0 [0–30]
Side (Left/Right)	(7), 33%/(14), 67%	(9), 43%/(12), 57%
Etiology		
Genetic	(8), 38%	(7), 33%
Unknown	(7), 33%	(11), 52%
Otosclerosis	(3), 14%	(1), 5%
Ménière's disease	(2), 10%	(1), 5%
Trauma	(1), 5%	(0)
Meningitis	(0)	(1), 5%

*Data are expressed as mean ± standard deviation [min–max], and (n), %*.

**Table 2:** Hearing outcomes according to electrode array insertion technique, array translocation, and distal (>180°) and proximal (<180°) translocations.

	**SDS**	**PTA**		
	**60 dB**	**Low-frequency**	**Mid-frequency**	**High-frequency**
**Insertion technique**				
Robot-assisted (21)	66 ± 30.8 [0–100]	30 ± 8.6 [19–48]	33 ± 11.2 [16–50]	42 ± 22.6 [13–110]
Manual (21)	65 ± 25.8 [0–100]	31 ± 9.9 [20–66]	33 ± 15.1 [23–92]	35 ± 21.6 [23–110]
**Position of the electrode array**				
No translocation (30)	69 ± 27.2 [0–100]	31 ± 10.1 [19–66]	33 ± 14.5 [16–91]	42 ± 23.8 [13–110]
Translocation (12)	58 ± 29.5 [0–90]	31 ± 6.5 [20–40]	33 ± 9.1 [18–51]	42 ± 17.1 [22–75]
**Localization of the translocation**				
Distal (4)	71 ± 14.3 [60–90]	27 ± 3.1 [25–32]	27 ± 4.8 [23–34]	28 ± 5.6 [25–36]
Proximal (8)	51 ± 33.5 [0–90]	33 ± 6.8 [20–40]	37 ± 9.3 [19–51]	49 ± 16.9 [22–75]^*^

*Data are expressed as mean ± SD [min–max]*.

*SDS: speech discrimination score at 60 dB in silence (%)*.

*PTA: pure-tone average (dB)*.

* *Comparison between distal and proximal translocation, p < 0.05 (Mann–Whitney test)*.

### Hearing Performance and the Hearing Loss Etiology

The speech perception at 1 year was similar according to the etiology of the hearing loss (*p* = 0.3; Kruskal-Wallis and Bonferroni *post-hoc* test). The translocation rate was not associated with the etiology of the hearing loss (*p* = 0.75; Chi-square and *post-hoc* pairwise comparisons; Table 3).

**Table 3:** Speech perception and array translocation according to the etiology of the hearing loss.

**Etiology**	**N**	**SDS 60 dB**	**Array translocations**
Unknown	18	57 ± 28.6	4 (22)
Genetic	15	74 ± 28.9	5 (33)
Otosclerosis	4	68 ± 28.7	2 (50)
Meniere's disease	3	81 ± 17.5	0 (0)
Meningitis	1	80	1 (100)
Traumatic	1	55	0 (0)

*SDS 60 dB: speech discrimination score at 60 dB in silence (%)*.

*The array translocation is expressed as the number of array translocation and the percentage by etiology: n (%)*.

### Hearing Performance and Intrascalar Position of the Electrode Array

Twelve array translocations (28%) were observed, and the translocation rate was similar whatever the type of electrode array (*p* = 0.09; Fisher's exact test). Moreover, the ratio of array translocation was similar in robot-assisted (*n* = 5, 24%), and manual (*n* = 7, 33%) insertion. However, considering the number of translocated electrodes, this was lower in the case of robot-assisted insertion (*n* = 34, 8.6%) compared to manual insertion (*n* = 56, 14%) (*p* = 0.018; CI 95%: =0.35–0.91; Fisher's exact test; Figure 2).

**Figure 2:** Representation of the position of each electrode following robot-assisted and manual electrode array insertion. The position of the electrode array was adjusted according to the round window position (RW) (dotted line) and 180° position (continuous line). The translocation rate of the electrode array was similar in both insertion groups, however, the number of translocated electrodes after a robot-assisted insertion was lower than with manual insertion. Unfilled circles: non-translocated electrode, filled circles: translocated electrode. AB, Advanced Bionics; * electrodes inserted through a cochleostomy.

Array translocation was not associated with an impaired speech perception in silence (translocation: 58 ± 29.5% *n* = 12; no translocation: 69 ± 27.2% *n* = 30; *p* = 0.23, Mann–Whitney test). With regard to pure tone audiometry, there were no differences between translocation and no translocation of the electrode and the low-frequency PTA (*p* = 0.62), mid-frequency PTA (*p* = 0.51), or high-frequency PTA (*p* = 0.53; Mann–Whitney test; Table 2). Considering the location of the translocation of the array, the high-frequency PTA was significantly better in distal than in proximal translocations (28 ± 5.6 dB, and 49 ± 16.9 dB, respectively; *p* = 0.04, Mann–Whitney test; Table 2).

Regarding the number of translocated electrodes, there was still no correlation between the percentage of translocated electrodes and speech performance in silence (*p* = 0.14; rho = −0.23; Spearman's rank correlation). This trend did not vary for the low-frequency PTA (*p* = 0.35; rho 0.15; Spearman's rank correlation), mid-frequency PTA (*p* = 0.34; rho = 0.15; Spearman's rank correlation), and high-frequency PTA (*p* = 0.40; rho = 0.13; Spearman's rank correlation).

In two cases (4%), the electrode was inserted through a cochleostomy (Figure 2). In both cases, the electrode array was translocated and had a poor speech perception (robot insertion-MS: 30% and manual insertion-CI522/622: 0%). Regarding the pure-tone audiometry thresholds, both cases had an increased high-frequency PTA (45 and 75 dB, respectively).

### Relationship Between Speech Perception in Silence and High-Frequency Thresholds in Pure-tone Audiometry

At 1 year post-implantation, the overall speech perception in silence with the implanted ear was improved: pre-implantation SDS: 0 ± 0%; post-implantation: manual: 65 ± 25.8% (*n* = 21), and post-implantation: robot-assisted: 66 ± 30.8% (*n* = 21). Neither low-frequency PTA nor mid-frequency PTA was associated with the speech perception scores (Figure 3). On the other hand, restoration of high-frequency thresholds was associated with better speech perception (fractional polynomial non-linear regression, *p* < 0.0001; Adjusted *R*^2^ = 0.64). Patients with speech perception scores > 50% clearly had better high-frequency PTA (36 ± 16.0 dB; *n* = 34) than those with speech perception scores ≤ 50% (76 ± 24.8 dB; *n* = 8) (*p* < 0.001; Mann–Whitney test). With regard to the electrode array type, the speech performance in silence was similar whatever the electrode array used (AB Mid-Scala: 70 ± 25.2%, *n* = 6; AB Slim J: 72 ± 27.6%, *n* = 16; CI522/622: 70 ± 30.0% *n* = 20; *p* = 0.92, Kruskal–Wallis test). The depth of insertion was not correlated with speech perception in silence (*p* = 0.52; rho = 0.10, Spearman's Rank correlation).

**Figure 3:** Speech perception at 60 dB in silence and pure-tone audiometry thresholds. The line represents a non-linear regression [*f*_(*x*)_ = 0.008x^2^-0.38x + 35.1, *p* < 0.0001; Adjusted *R*^2^ = 0.64], and the gray zone represents the 95% confidence interval. The area within the dotted lines indicates a poor speech perception lower than 50% and a high-frequency PTA higher than 50 dB. Triangles: robot-assisted insertion; circles: manual insertion; filled symbols: translocation of the electrode array; unfilled symbols: non-translocation.

## Discussion

In this preliminary study, hearing outcomes after robot-assisted or manual array insertion were evaluated 1 year after cochlear implantation. Regardless the electrode array insertion technique, speech perception in silence was improved when the pure tone thresholds at high frequencies were restored after cochlear implantation. In the case of translocation of the electrode array, robot-assisted insertion reduced the number of translocated electrodes compared with manual insertion, but this was not related to an improvement in speech perception in silence.

Although the association between speech perception in silence and high-frequency thresholds in pure-tone audiometry has not been reported in cochlear-implanted patients, previous reports showed the association of speech perception in non-implanted patients with hearing loss, especially at high frequencies (15, 18). Another study, in non-implanted patients, showed the importance of preservation of the extended high frequencies (>8,000 Hz) and the performance in noise (19). Our findings are in agreement with an earlier study showing no correlation between speech perception and PTA (125–8,000 Hz) in cochlear-implanted patients (13). Another study reported five patients successfully implanted with the RobOtol® and a restoration of frequencies from 250 to 4,000 Hz; however, its association with speech perception was not analyzed (9). Regarding the electroacoustic stimulation of cochlear implant candidates, the improvement in hearing performance was focused on preservation of the low-frequency range (5, 20). However, the spectral range of voice, which includes vowels and consonants, could involve a wider frequency range from 200 to 10,000 Hz for fricative consonants such as “s” or “f” (21). As the cochlear ramp is tonotopically arranged and due to the characteristics of the electrode array, merely medium and high frequencies could be stimulated and restored.

Our results showed similar hearing outcomes for speech perception in silence and pure-tone audiometry thresholds with robot and manual electrode array insertions. This could be explained by the fact that the robot was entirely handled by the surgeon according to its mental representation of the cochlear structures. Earlier studies reported the importance of inserting the electrode array along the optimal axis to reduce intracochlear trauma (11). In addition, for pre-curved arrays such as the Mid-Scala, alignment of the array tip with the coiling direction of the scala tympani could be a critical step to reduce intracochlear trauma (12). The alignment of the array with the insertion axis could be similar to manual insertion or using the RobOtol®, because in both insertion techniques, the surgeon had no visual information to correctly determine the optimal axis of insertion. However, the advantages of using the RobOtol® are to insert the electrode array in a smooth way, to decompose motion into pure rotation or translation and to eliminate the involuntary movements of the hand such as tremor, all these movements are very difficult to perform manually. The next step could be accomplished by coupling the robot and navigation to insert the electrode array in the most appropriate way. A personalization of the array insertion would aim to reduce the intracochlear trauma according to the anatomy of the patients and the surgical circumstances such as inserting the electrode array in the optimal axis (11), align the array with the coiling direction of the ST specifically for the pre-curved electrodes (12), and adapting the insertion through the round window or a cochleostomy considering the hook region of the cochlea (22). Likewise, future investigation should be focused to have a haptic feedback, control the direction of the array with steering tools, and/or have an intracochlear visualization during the array insertion.

Our results are in contrast to earlier studies showing worse speech performance when translocation of the electrode array was observed (2, 3, 23, 24). We performed a detailed analysis of the position of the electrode array to determine the intrascalar position of each electrode, and our findings are in contrast to previous reports that showed an association between an array fully inserted into the scala tympani and better speech performance (1–3). Regarding the localization of the translocation, a proximal translocation was associated with a decrease in high-frequency PTA. This decrease could be due to the fact that high-frequencies are delivered to the spiral ganglion by the proximal electrodes. Although a decrease in the high-frequency thresholds would be more deleterious for speech perception, no difference was observed between proximal and distal translocation.

The electrode array position was reconstructed and evaluated from the postoperative CT imaging made in the first 24 h. Previous studies showed that a migration (25) or an extrusion of the electrode array is a complication that could be suspect when a gradual increase of the impedances is observed (26). In our study, there was no assessed a slight migration of the electrode array, however a postoperative CT scan was performed in case of an unexplained degradation or a persistence of poor hearing performance. Thus, no extrusion of the electrode array was detected in our series.

The study has some limitations. First: the groups (robot-assisted and manual insertion) were paired by age, duration of profound deafness and electrode array type. However, we cannot exclude variability due to the etiology of hearing loss. Second: the sampling method was taken in a non-probability way (hearing performance at 1 year of the first patients implanted by the robot). A randomized study would be required to compare the hearing performance of the robot-assisted array insertion to manual ones.

In summary, this is a preliminary study to provide hearing outcomes for robot-assisted electrode array insertion. Regardless the array insertion technique (robot-assisted or manual), our data suggest that restoration of high frequency thresholds (3,000–4,000–8,000 Hz) is associated with better speech perception in silence 1 year postoperatively. The intrascalar position of the array was not associated with hearing performance but proximal translocation was deleterious to high frequency thresholds. A prospective and randomized trial with comparable groups will be required to assess the relevance of robot-based insertion in hearing performance.

## Data Availability Statement

The raw data supporting the conclusions of this article will be made available by the authors, without undue reservation.

## Ethics Statement

The studies involving human participants were reviewed and approved by CNIL N° 20191219182243. The patients/participants provided their written informed consent to participate in this study.

## Author Contributions

RT, HD, GL, OS, EF, IM, and YN contributed to conception and design of the study. RT and HD organized the database. RT performed the statistical analysis and wrote the first draft of the manuscript. All authors contributed to manuscript revision, read, and approved the submitted version.

## Funding

The study was supported by research funding from Fondation pour l'Audition (Starting Grant IDA-2020), ANR Robocop ANR-19-CE19-0026-02.

## Conflict of Interest

The authors declare that the research was conducted in the absence of any commercial or financial relationships that could be construed as a potential conflict of interest.

## Publisher's Note

All claims expressed in this article are solely those of the authors and do not necessarily represent those of their affiliated organizations, or those of the publisher, the editors and the reviewers. Any product that may be evaluated in this article, or claim that may be made by its manufacturer, is not guaranteed or endorsed by the publisher.
